The article "Analysis of the Preventive Action of Rivaroxaban against Lower Extremity Deep Venous Thrombosis in Patients after Laparoscopic Radical Gastrectomy" was published in 2022. Journal: Comput Math Methods Med.

# Analysis of the Preventive Action of Rivaroxaban against Lower Extremity Deep Venous Thrombosis in Patients after Laparoscopic Radical Gastrectomy

**DOI:** 10.1155/2022/7140066

**Published:** 2022-09-10

**Authors:** Qinhui Dong, Xiayin Zhu, Yafen Gao, Zhengrong Wang, Dexing Zheng, Jian Zhu

**Affiliations:** ^1^Derpartment of Medical Oncology, Taizhou Hospital of Zhejiang Province Affiliated to Wenzhou Medical University, Linhai, 317000 Zhejiang, China; ^2^Derpartment of Hematology, Taizhou Hospital of Zhejiang Province Affiliated to Wenzhou Medical University, Linhai, 317000 Zhejiang, China; ^3^Derpartment of Vascular Surgery, Taizhou Hospital of Zhejiang Province Affiliated to Wenzhou Medical University, Linhai, 317000 Zhejiang, China; ^4^Derpartment of Radiotherapy, Taizhou Hospital of Zhejiang Province Affiliated to Wenzhou Medical University, Linhai, 317000 Zhejiang, China

## Abstract

**Background:**

Gastric carcinoma (GC) is a common lethal cancer in the world. Patients are prone to develop lower extremity deep venous thrombosis (LEDVT) after laparoscopic radical gastrectomy (LRG), which threatens their life and health.

**Purpose:**

This research is to clarify the preventive action of rivaroxaban (Riv) against LEDVT in patients undergoing LRG.

**Methods:**

A retrospective study was conducted on 70 patients with GC admitted for LRG between January 2019 and January 2022, including 40 patients (observation group) receiving Riv treatment and 30 patients (conventional group) treated with air wave pressure therapy apparatus. Quality of life, coagulation function, LEDVT formation, and complications were compared between groups.

**Results:**

The observation group had better recovery of life quality than the control group, along with more effective inhibition of coagulation disorders, less DVT formation, and fewer complications.

**Conclusions:**

Compared with air wave pressure therapy apparatus, Riv has better preventive action against LEDVT in GC patients after LRG.

## 1. Introduction

As far as the influence of gastric carcinoma (GC) on the global population is concerned, it ranks fifth in prevalence among cancers and third in cancer-related mortality [1, 2]. Various factors, including smoking, drinking, Helicobacter pylori infection, and high salt, oil, and sugar food intake, will increase the risk of GC [3–5]. Clinically, open surgery is the major approach to treat gastric adenocarcinoma, but it is prone to cause greater harm to patients [6]. In recent years, laparoscopic surgery, a procedure less invasive with milder postoperative pain and faster recovery than open surgery, has become increasingly common [7]. However, the complexity of laparoscopic surgery for GC, improper operation of medical staff during surgery, and patient insufficient compliance can easily lead to accidents, so how to prevent all kinds of complications after surgery is critical [8, 9].

Venous thrombosis of the lower extremities is the most common adverse event after laparoscopic treatment [10]. DVT occurs when a blood clot forms in the vein of the leg. The thrombus can even rupture and travel to the lungs, resulting in potentially severe blood flow obstruction (pulmonary embolism or PE) or even death [11]. In the lower extremities, the primary route of venous blood flow is the deep vein rather than the superficial vein. As a result, DVT causes impaired venous return of the lower extremities, resulting in limb swelling, discomfort, and gait disturbance. It is reported that nearly 2.5 to 5 percent of the population are affected by DVT at some stage in their lives [12]. Although anticoagulant therapy is widely available for the disease, more than half of patients develop postthrombotic syndrome within two years of DVT, characterized by leg pain, swelling, skin pigmentation, or venous ulcers [13, 14]. In this study, we will take rivaroxaban (Riv) as an example to explore its preventive action against lower extremity deep venous thrombosis (LEDVT) of patients after laparoscopic radical gastrectomy (LRG).

## 2. Methods

### 2.1. General Information

Seventy patients admitted and underwent LRG between January 2019 and January 2022 were selected and assigned to a control group with 30 cases and an observation group with 40 cases. The general data of the two cohorts were comparable with no statistical differences.

Patients meeting the following criteria were enrolled: ① in accordance with the World Health Organization (WHO) tumor diagnostic criteria established in the Pathology and Genetics of Tumors of the Digestive System [15], with surgical tolerance; ② preoperative diagnosis of LEDVT [16] by vascular ultrasonography; and ③ adults (age > 18). Patients were excluded according to the following criteria: ① recent active bleeding, ② blood system-related diseases or coagulopathy, ③ use of anticoagulant drugs because of other diseases, and ④ presence of LEDVT before operation.

Patients and their families were informed of this study and all signed informed consent. The Medical Ethics Committee approved the study protocol without reserves, and this study was conducted strictly following the Declaration of Helsinki.

### 2.2. Methods

Both groups of patients underwent LRG under general anesthesia, which was performed by the same surgical team. No hemostatics were used postoperatively. The next day after surgery, patients were instructed to ambulate to exercise their ankles, toes, knees, and other joints. In the control group, air wave pressure therapy apparatus was used to prevent LEDVT. The medical staff assisted the patient to wear the multichamber airbag leg sleeve and set the time as 30 min. The first use of the instrument followed the principle of gradually increasing the pressure, so that patients could gradually get used to it and wear it for a longer duration. The maximum tolerable pressure was determined according to patients' feelings. The observation group was given Riv (Bayer Pharmaceuticals, approval number: H20100464, specification 10 mg/tablet) for thrombosis prophylaxis, which was administrated orally, 10 mg/time, once daily, for 10 days.

### 2.3. Outcome Measures

#### 2.3.1. Postoperative Quality of Life (QoL)

The postoperative life status of the two cohorts was observed and compared from the aspects of sleep status and activities of daily living (ADL). The sleep quality assessment used the Pittsburgh Sleep Quality Index (PSQI, score range: 0-21) [17], with the score in inverse proportion to the sleep quality and a score greater than 7 indicating sleep disorders. As to the ADL, it was evaluated with the activity of daily living scale [18], an instrument with a score range of 0-100. The score is negatively related to self-care ability, and a score less than 60 points means that the patient needs help in life.

#### 2.3.2. Coagulation function

Patients' venous blood was collected before and 10 days after surgery to measure the changes of fibrinogen (Fbg), activated partial thromboplastin time (APTT), prothrombin time (PT), and thrombin time (TT) using the LHOTSYS series automatic biochemical analyzer (approval number: Guangdong Food and Drug Supervision Machinery Zi 2012 no. 2400609, manufacturer: Shenzhen Glory Medical Co., Ltd., specification: BS-3600 T).

#### 2.3.3. DVT Formation

DVT formation of patients, which was mainly judged by lower limb temperature, skin color, and swelling, was recorded and compared. For those with abnormalities and highly suspected DVT formation, immediate physical examination and color Doppler ultrasonography of the lower extremities were performed. Color Doppler ultrasonography diagnosis criteria for DVT are as follows: significant substantial echo in the lumen of lower limbs, no voluntary blood flow at the thrombus, and failure to deflate the patient's veins.

#### 2.3.4. Complication Rate

The postoperative complications of the two groups were compared. The associated indicators included nausea, vomiting, labored breathing, and chills.

Among the above indicators, PSQI and activity of daily living scale scores, coagulation function-related indicators (Fbg, APTT, PT, and TT), and incidence of DVT were the primary outcome measures, while the incidence of complications such as nausea, vomiting, labored breathing, and chills were the secondary ones.

### 2.4. Statistical Methods

Integrated data processing was done by SPSS 22.0 (Asia Analytics Formerly SPSS China). The statistical method for categorical data (denoted by *n* (%)) was *χ*^2^; quantitative data, denoted by *X* ± *S*, were analyzed by *t*-test or pair *t*-test (before and after surgery). *P* < 0.05 was the significance level for all analyses.

## 3. Results

### 3.1. General Information

The two cohorts showed no statistical difference in sex, age, body mass index (BMI), tumor node metastasis (TNM) staging, and other general data (*P* > 0.05), see Table 1 for details.

### 3.2. Postoperative QoL

The comparison of patients' postoperative QoL revealed a lower PSQI score and a higher ADL score in the observation group compared with the control group, with statistical significance (*P* < 0.05, Figure 1).

### 3.3. Coagulation Function

Comparing patients' coagulation function, it was found that APTT, PT, and TT were significantly higher and Fbg was lower in the observation group, versus the control group, with statistical significance (*P* < 0.05, Figure 2).

### 3.4. DVT Formation

The intergroup comparison of DVT formation (Table 2) showed a lower overall incidence of DVT in the observation group (*P* < 0.05).

### 3.5. Complication Rate

The observation group had a statistical lower complication rate than the control group, as indicated by intergroup comparison data of the incidence of complications displayed in Table 3 (*P* < 0.05).

## 4. Discussion

Early diagnosis and treatment of GC, a highly lethal and recurrent tumor worldwide, is crucial [19]. Laparoscopic resection has recently become a common treatment for GC, but there are still many problems caused by misoperation [20–22]. After laparoscopic surgery, the incidence of DVT increases, and postthrombotic syndrome can exert a long lasting effect on the patients' daily life [23]. Therefore, DVT prophylaxis is necessary. This study mainly discusses the preventive action of Riv against postoperative thrombosis after LRG from two aspects: coagulation function and postoperative recovery.

In terms of coagulation function, the observation group using Riv was observed with an obviously better coagulation function than the control group. Riv, as a standard coagulation inhibitor, has an inhibiting effect on factor Xa and plays a vital part in various thromboembolic and atherothrombotic diseases [24]. Factor Xa is essential in both intrinsic and extrinsic coagulation pathways that lead to downstream thrombin activation and clot formation [25], while Riv can reversely inhibit small molecules of the free and clot-bound factor Xa. Due to this function, Riv is not only increasingly used in various vascular diseases (coronary artery diseases, peripheral artery diseases, and thrombosis prophylaxis in particular) but also applied to the treatment of nonvalvular atrial fibrillation and DVT or venous embolism [26]. Another preventive measure, air wave pressure therapy apparatus, is often used to prevent DVT due to its ability to remove thrombosis directly by compression. However, if DVT is found to exist in lower limbs upon admission, improper prevention and control of DVT with air wave pressure therapy apparatus may induce thrombosis displacement, which may lead to PE [27]. This study showed better coagulation function in the observation group due to the use of Riv that can dissolve thrombus in a molecular mechanism. Therefore, compared with the control group which only used air wave pressure therapy apparatus to break thrombus, the coagulation function of the observation group was not significantly inhibited. Take Fbg as an example, as a glycoprotein complex, Fbg is enzymatically converted into fibrin by thrombin during tissue injury, causing blood to clot and stop bleeding. A clinical study on coronavirus disease 2019 (COVID-19) found a prothrombic diathesis in critical COVID-19 patients with significantly high Fbg levels, as well as higher Fbg levels [28]. Combining the above with our findings, we can find that compared with the control group which prevented thrombosis by compression, the observation group has lower Fbg level and less DVT formation due to the effective reduction of coagulation disorders in the molecular mechanism. In the retrospective study of Zhang et al. [29], Riv was applied to patients with severe craniocerebral injury after surgery, which also had an effective prevention effect on postoperative DVT, similar to our findings. In addition, Riv is reported to not only reduce the risk of recurrent venous thromboembolism but also have a certain preventive effect on postthrombotic syndrome [30].

When investigating patients' QoL and complications, we found that their sleep quality and life quality were effectively improved, and the incidence of complications was reduced. Consistently, Rashki Kemmak et al. reported that Riv intervention can reduce medical costs while significantly improving the QoL of patients undergoing total knee or hip arthroplasty [31]. Also, Becattini et al. [32] pointed out that Riv reduced the adverse events of patients after laparoscopic cancer surgery by 60% compared with placebo, which was consistent with our results. Thrombosis after surgery for various types of cancer has been reported in all major clinical manifestations with a significant negative impact on patient outcomes. Both proximal and distal PE can occur after DVT [33]. To make matters worse, cancer patients will have a poor prognosis and similar symptoms after thrombosis in either deep or superficial veins [34]. As a common complication after various operations, the formation of venous thromboembolism will have a certain impact on the postoperative QoL of patients [35]. Combining these, we can find that patients in the observation group treated with Riv had a faster recovery of QoL after surgery and were safer than those in the control group due to better outcomes.

The novelty of this study lies in the following: (1) The clinical effectiveness of Riv in patients after LRG was confirmed from the perspectives of PSQI and ADL scores and coagulation function-related indicators (APTT, PT, TT, and Fbg), demonstrating that it can significantly improve patients' QoL and coagulation function. (2) From the perspective of safety, it was confirmed that Riv had a significant preventive effect on LEDVT as well as other complications in GC patients after LRG. However, there are still many deficiencies in this study. For example, we had not investigated patients' satisfaction at discharge, which is one of the defects of this study. In future experiments, we will address it and continue to improve the treatment plan, so as to make patients more satisfied. Besides, we should detect more targeted molecules or inflammatory factors related to GC, to better monitor the recovery of patients.

## 5. Conclusion

Conclusively, compared with air wave pressure therapy apparatus, Riv is more effective in preventing LEDVT in patients after LRG, which is worthy of further clinical promotion.

## Figures and Tables

**Figure 1:** Postoperative quality of life. (a) PSQI score: an obviously lower PSQI score was determined in the observation group compared with the control group (*P* < 0.05). (b) ADL score: an obviously higher ADL score was determined in the observation group compared with the control group (*P* < 0.05). Note: compared with the control group, ^∗^*P* < 0.05.

**Figure 2:** Coagulation function. (a) Fbg: significantly changed Fbg was observed in both cohorts after surgery, with a higher level in the control group as compared to the observation group (*P* < 0.05). (b) APTT: significantly changed APTT was observed in both cohorts after surgery, with a higher value in the observation group as compared to the control group (*P* < 0.05). (c) PT: markedly changed PT was observed in both cohorts after surgery, with a higher value in the observation group as compared to the control group (*P* < 0.05). (d) TT: markedly changed TT was observed in both cohorts after surgery, with a higher value in the observation group as compared to the control group (*P* < 0.05). Note: ^∗^*P* < 0.05, compared with the control group and ^#^*P* < 0.05, compared with the posttreatment value.

**Table 1:** General data.

Classification	Observation group (*n* = 40)	Control group (*n* = 30)	*t*/*χ*^2^	*P*
Sex			0.33	0.568
Male	24 (60.00)	20 (66.67)		
Female	16 (40.00)	10 (33.33)		
Age (years old)	58.18 ± 6.46	58.50 ± 7.62	0.190	0.850
BMI (kg/m^2^)	22.88 ± 1.18	23.23 ± 1.04	1.291	0.201
TNM staging			0.02	0.890
II	22 (55.00)	17 (56.67)		
III	18 (45.00)	13 (43.33)		
Operation plan			0.08	0.777
Total gastrectomy	16 (40.00)	11 (36.67)		
Distal gastrectomy	24 (60.00)	19 (63.33)		
Drinking			0.03	0.872
Yes	30 (75.00)	23 (76.67)		
No	10 (25.00)	7 (23.33)		
Eating habits				
Heavy	32 (80.00)	21 (70.00)	0.93	0.334
Light	8 (20.00)	9 (30.00)		

**Table 2:** DVT formation in the two groups.

	Observation group (*n* = 40)	Control group (*n* = 30)	*χ* ^2^	*P*
Postoperative DVT	1	6	—	—
Total incidence (%)	2.50	20.00	5.83	0.016

**Table 3:** Incidence of complications in two groups of patients.

	Observation group (*n* = 40)	Control group (*n* = 30)	*χ* ^2^	*P*
Nausea	1 (2.50)	0 (0.00)	—	—
Vomiting	0 (0.00)	6 (20.00)	—	—
Labored breathing	0 (0.00)	3 (10.00)	—	—
Chills	1 (2.50)	0 (0.00)		
Incidence rate of complications	2 (5.00)	9 (30.00)	8.09	0.005

## Data Availability

The labeled datasets used to support the findings of this study are available from the corresponding author upon request.
